RETRACTED

# Gut Microbiota Profiles in Dairy Cattle from Highland and Coastal Regions Using Shotgun Metagenomic Approach

**DOI:** 10.1155/2022/3659052

**Published:** 2022-09-09

**Authors:** Bambang Waluyo Hadi Eko Prasetiyono, Widiyanto Widiyanto, Nuruliarizki Shinta Pandupuspitasari

**Affiliations:** ^1^Laboratory of Feed Technology, Animal Science Department, Faculty of Animal and Agricultural Sciences, Universitas Diponegoro, Indonesia; ^2^Laboratory of Animal Nutrition and Feed Science, Animal Science Department, Faculty of Animal and Agricultural Sciences, Universitas Diponegoro, Indonesia

## Abstract

There is significant difference in milk production of highland and coastal regions in Indonesia of which the latter is critically low. The recent studies indicate a possibility of improving the milk yield and quality by manipulating the gut microbiota, for which profiling and abundance of gut microbiota in these divergent regions need to be addressed. The present study was the first of its kind to explore the dairy cattle gut microbiota diversity, abundance, and functional annotation of the two divergent Indonesian regions, the highland and coastal regions, by shotgun metagenomic approach. Unfavorable environmental conditions such as type of forage grass in coastal regions and high temperature remain a limiting factor; however, the improvement through manipulating the gut microbiota was not considered until recently to improve the quality and quantity of coastal region dairy cattle. The application of recent advance technologies can help achieve this goal on sustainable basis. The results show Bacteroidetes in higher abundance in coastal region (FPP) than in highland (Salatiga) while Firmicutes were higher in Salatiga. Furthermore, a collective physiology of the community was found by annotating the sequences against KEGG, eggNOG, and CAZy databases. To identify the role in pathways, an mPATH analysis was performed to have insight into the microbiota community in different metabolic pathways. The identified targets can be used as prebiotic and/or probiotic to improve the average milk yield of coastal region dairy cattle by manipulating the dairy feed with desired microbes.

## 1. Introduction

Indonesian dairy industry production remains at 1,800 tonnes of milk a day in 2022 which only provides 5% of the country demand [1]. The average daily production by local farmers in Indonesia ranges from 4 to 6 litters a day while the Holstein cow production varies 16-20 litters a day which is much lower than its potential [2]. However, it was observed that highland dairy cattle produced 45 litters of milk on average in comparison to coastal region dairy cows.

The gut microbiota of cow and its abundance are associated with a wide range of activities and functions such as fermentation of feed, fatty acid formation, methane production, nitrogen emissions, and cellulose digestion [3]. The cow's rumen houses ancestrally diverse community of anaerobic bacteria, viruses, ciliated protozoa, fungi, and methanogenic archaea. These microbiota are capable of degrading indigestible plant fibre of the host [4, 5]. The rumen microbiome is critical for the host animal's nutrition, by providing essential nutrients by fermentation of feed, which on ruminant growth in number of ways. The ruminants especially dairy cows are dependendent on the microbial metabolites for the production of economically important products such as milk.

RETRACTED

The most convoluted microbial communities which inhabit the rumen have triggered the microbiologists' curiosity. Physiologists and nutritionists are also aware of the rumen's critical role in the digestion of fibrous feed and the provision of the host animals' nutritional requirements. They enable the ruminants to provide food to people [6]. Furthermore, as previously demonstrated by a relationship between microbiome components and residual feed intake, the composition of these various types of microbes influences the productive efficiency [7, 8].

The composition of the rumen microbiota has been widely studied previously across various regions of the globe for various reasons [9]. Microbes work alongside the host to provide them with their metabolic products [10]. Ciliate protozoa account for 50% of microbial community of the cow gut [11]. The protozoa also vary greatly in ruminants in terms of abundance or diversity, but their presence or absence is not greatly impactful to the host as a great amount of their products can also be synthesized by other groups of the gut microbiota [9, 12].

Anaerobic fungi break down plant's toughest structure for efficient usage of feed [13]. In CH4, the Archaea are important contributors [14, 15]. Several studies have been done on dairy cow's gut microbiota for their roles in various pathways and metabolic activities [16–19], where recently heritable component of the gut microbiota are reported [20]. Microbiota are composed mainly of bacterial families along with Archaea and fungi, each of them working to produce various important compounds for the host [21, 22]. It is also extensively studied that the type and colony size of these microbiota are effected by factors such as temperature, pH, feed, water quality, age, genetics, region, and health [23–25].

Several factors including age, diet, genetics, and feed efficiency and environmental stimuli affect the rumen microbiota composition which directly influence the productivity of host [26]. The present study was an effort to explore the fecal gut microbiota of the highland and coastal region dairy cattle in Indonesia to explore its abundance and to figure out the potential prebiotic and probiotic candidates to enhance quantity and quality of the coastal region dairy cattle in Indonesia.

RETRACTED

## 2. Material and Methods

### 2.1. Farm and Animal Selection

The well managed farms which keep the organized record of dairy cattle in highland and coastal areas of Indonesia were selected for the study. The fecal samples of healthy cows were collected in DNA/RNA shield tubes. The DNA/RNA shield tubes were brought back to laboratory for further processing. DNA was extracted from the fecal samples utilizing 1 gram of the collected sample [27]. The quality test for the extracted DNA sample was performed before constructing libraries for the samples.

For library construction, genomic DNA was sheared randomly into short fragments. The fragments obtained were A-tailed and end repaired and then ligated to Illumina adapter. The adapter-ligated fragments were amplified using PCR, selected for size, and then purified. Qubit was used to check library for quantification by real-time PCR, and the bioanalyzer was used to detect size distribution. The libraries that were quantified were pooled, and Illumina platforms were used to sequence, as per the requirements of the effective library concentration and the amount of data required.

### 2.2. Bioinformatic Analysis

The certain percentage of low-quality data reads obtained in raw data after sequencing was host filtered to establish the accuracy and reliability of the subsequent information analysis to obtain effective data termed as clean data; clean data was used to assemble metagenome after quality control of each sample, and mixed assembly was made from unutilized reads to explore the information regarding low abundant species from each sample. MetaGeneMark was used for the gene prediction utilizing scaftigs which were assembled by single and mixed samples. Gene catalogue was constructed by pooling the predicted genes for dereplication. The abundance information of each sample was obtained from the gene catalogue. Metagenomic reads were compared to NR database, i.e., the database of taxonomically informative gene families for annotation of each metagenomic homolog. Gene abundance table was obtained from the abundance tables of different taxonomic ranks. The coding sequence function was obtained from its similarity to sequences in three databases, i.e., KEGG, eggNOG, and CAZy. Doing this for all metagenomic sequences, we produced a profile of distinct types of functions and their relative abundance in the studied metagenome.

RETRACTED

## 3. Results and Discussion

The next generation sequencing (NGS) was used to obtain the sequencing reads from metagenomic DNA isolated from fecal samples of coastal region (FPP) and highland (Salatiga) dairy cattle. The sequencing was done on NovoSeq6000. The sample coastal region (FPP) and highland (Salatiga) produced 7.15 GB and 7.33 GB of raw base data, respectively. The clean bases for coastal region (FPP) and highland (Salatiga) were 7.14 GB and 7.33 GB of raw bases, respectively. The data with less than 0.001 sequencing error rate in coastal region (FPP) and highland (Salatiga), i.e., Clean_Q30, were 94.72% and 94.02%,, respectively. In all the assembled results, all scaftigs were counted and the distribution of scaftigs length in each sample. A mixed assembly was conducted on the reads that were unutilized keeping the same assemble parameter. The results are presented in Figure 1.

### 3.1. Taxonomic Analysis of Highland and Coastal Region Dairy Cattle

The question of communities' similarity needs to be ascertained by identifying reads that serves as the marker gene homologs to a taxonomically informative gene families by phylogenetic and sequence similarity to NR database [28] and to annotate taxonomically each metagenomic homolog (MEGAN [29]). Several analyses were performed according to abundance table at each taxonomic level.

### 3.2. Relative Abundance of Bacteria in Highland (Salatiga) and Coastal (FPP) Farms

As reviewed earlier, the milk yield in coastal regions is critically low. To identify the reasons behind this low milk yield, we compare the gut microbiota of highland to coastal region dairy cattle. We found that Bacteroidetes were at higher abundance, i.e., 52% in coastal region to that of 37% in highland. Bacteroidetes is a phyla that is mostly producing metabolites that are responsible for hormones that causes satiety and weight loss [30, 31]. As we observed, the dysbiosis of Bacteroidetes in coastal region indicates that it might be one of the reasons for lower milk yield in coastal region.

Furthermore, the data indicate that the Prevotella sp. MGM2 was highly abundant in coastal region, i.e., 19% to 2% in highland region. It has been identified that Prevotella sp. MGM2 is involved in enhancing Treg cells which is an indication of poor health of host [32]. The Prevotella sp. CAG:891 shows 11% in coastal region and 3% in highland region. Prevotella sp. CAG:891 is responsible producing L-pipecolic acid of which higher concentrations are associated with metabolic disorders [33].

It is noteworthy that the abundance of Prevotella sp. CAG:485 shows lower abundance, i.e., 0.6% in coastal region to that of 5% in highland region. Prevotella sp. CAG:485 produces metabolite grpE which participates in active response to hyperosmotic pressure and heat stress [34]. It prevents the accumulation of unfolded proteins in the cytoplasm and hence provide protection against death. The lower abundance in coastal region (FPP) is indicating the lesser ability coastal dairy cattle of lesser ability to resist heat and higher temperature which negatively affects milk yield and quality (Figure 2).

RETRACTED

### 3.3. Functional Annotation of Coastal and Highland Dairy Cattle Fecal Gut Microbiota

The identified unigene functional annotation was performed against the CAZy [35], eggNOG [36], and KEGG [37] databases, and the results obtained are shown in Figures 3(a)–3(c). We observed that coastal region (FPP) dairy cattle showed statistically significant higher number of pathway genes for metabolism, environmental information processing, cellular processes, and genetic information processing. Scientifically, dairy cattle shows that higher metabolic rate produces lower quantity of milk.

The eggNOG database revealed several pathway genes related to metabolism including nucleotide transport and metabolism, amino acid transport and metabolism, coenzyme transport and metabolism, carbohydrate transport and metabolism, inorganic ion transport and metabolism, and lipid transport and metabolism (Figure 3(c)). The significant unigene number involved with metabolism is 2163, cellular processes is 210, and environmental information processing is 188 as shown in Figure 3(d). The CAZy database shows a large number of glycoside hydrolases and glycosyl hydrolases (Figure 3(b)).

### 3.4. Metabolic Pathway

To further elaborate metabolic pathways among samples, we apply mPATH analysis. We created a web version pathway report which demonstrates variances of pathway patterns. We obtained shared and unique pathway information.

We identified that genes involved in uric acid cycle that may cause citrullinemia; i.e., disturbance in urea cycle was found to be unique for its expression in coastal region (FPP) dairy cattle.  Figure 4 shows the shared and unique pathway information for 2-oxycarboxylic acid metabolism. The data suggests if the dysbiosis in the gut microbiota of coastal region dairy cattle can be corrected will be way forward for high yielding and sustainable milk productions in future.

## 4. Conclusion

The high quality and quantity of milk yield are the desirable traits for dairy farming. The achievement of these traits is challenged by several factors including environmental stresses, diseases, and parasites. The animals do develop strategies to cope with such conditions; however, interventions to improve it accelerate the process. The use of advanced next generation sequencing technologies has brought an immense and targeted improvements in desired traits. The present study has explored the gut microbiota of coastal region (FPP) and highland (Salatiga) dairy cattle and found interesting targeted microbial species which after further validation can be developed as novel prebiotic and/or probiotic to improve milk quality and quantity specifically in coastal regions which can bring huge benefit to local farms of the coastal region in Indonesia.

RETRACTED

## Figures and Tables

**Figure 1:** Length distribution of scaftigs of different samples. The distribution of scaftigs length is calculated and plotted in each sample; frequency(#) is shown at the longitudinal axis; the number of scaftigs and the percentage of scaftigs number percentage (%) are represented in yellow curve. The scaftigs length is shown horizontally. (a) Sample coastal region (FPP). (b) Sample highland region (Salatiga). (c) NOVO-MIX.

**Figure 2:** Relative abundance in phylum and genus level in highland (Salatiga) and coastal regions (FPP): (a) phylum level; (b) genus level.

**Figure 3:** Relative abundance of each database. (a) KEGG unique gene level 1. (b) eggNOG unique gene level 1. (c) CAZy unique gene level 1. Summarized chart for the gene number annotated by every database: (d) KEGG pathway annotation; (e) eggNOG database; (f) CAZy database.

**Figure 4:** The compare analysis for oxocarboxylic metabolic pathway.

## Data Availability

Data can be requested to the corresponding author with a reasonable request.
